The article "Application Effect of Motion Capture Technology in Basketball Resistance Training and Shooting Hit Rate in Immersive Virtual Reality Environment" was published in 2022. Journal: Comput Intell Neurosci.

# Application Effect of Motion Capture Technology in Basketball Resistance Training and Shooting Hit Rate in Immersive Virtual Reality Environment

**DOI:** 10.1155/2022/4584980

**Published:** 2022-06-24

**Authors:** Wenting Wei, Ziqi Qin, Bihong Yan, Qiulin Wang

**Affiliations:** ^1^Physical Education Institute, Kunming University, Kunming 650000, Yunnan, China; ^2^Baita Middle School Panlong District Kunming, Kunming 650011, Yunnan, China; ^3^Physical Education Institute, Yangzhou University, Yangzhou 225000, Jiangsu, China

## Abstract

With the progress of society, sports have become the mainstream of social development. Strengthening the athletic ability of basketball players can effectively improve their shooting percentage. Firstly, virtual reality (VR) technology and motion capture technology are summarized. Secondly, the resistance training and shooting training of basketball players are analyzed and explained. Finally, the algorithm of motion capture technology is designed to capture and optimize the movements of athletes. In addition, a comprehensive evaluation of the shooting percentage of basketball players is carried out. The results show that the motion capture technology proposed here effectively captures the shooting action of basketball players, and the shooting percentage of players is promoted through resistance training. Among all athletes, the highest shooting percentage improvement is around 14% and the lowest is around 4%. In all groups, athletes of different heights have the largest difference in the improvement of shooting percentage. Therefore, this work plays an important role in improving the shooting rate of basketball players through VR technology. It provides technical support for improving the shooting percentage of basketball players and contributes to the progress of athletes' comprehensive athletic ability.

## 1. Introduction

More and more science and technology provide important support for human development [1]. Virtual reality (VR) technology is an advanced technology. It creates a virtual environment that is highly close to the real environment, thereby promoting the development of society [2]. Basketball is a popular sport at present. The main development direction of VR technology is to continuously improve the comprehensive athletic ability of basketball players [3]. Therefore, it is innovative to improve the comprehensive ability of basketball players through VR technology, and significant results can be achieved [4]. Although this technology is not yet mature, many studies have provided technical support for it.

Shao et al. pointed out that VR technology was an advanced human-computer interaction technology that effectively simulated human behaviors such as seeing, hearing, and moving in natural environments. It is the integration of artificial intelligence, computer graphics, human-machine interface technology, multimedia technology, network technology, parallel computing technology, and other technologies. This technology had been widely used in scientific visualization, flight simulation, medicine, remote sensing and remote control, education, entertainment, and other fields. With the continuous development of VR technology, it would show a broader application prospect. Therefore, introducing the research and development status of VR technology and popularizing VR technology were significant to promote the research and application of VR technology [5]. Baker et al. proposed that VR is a new human-computer interaction technology. It used a computer to generate a virtual environment and made the operator “immerse” into the environment through various sensing devices to realize the direct natural interaction between the operator and the environment. The virtual environment proposed here is a three-dimensional graphic generated by a computer, which could be a representation of a specific real environment in the real world or a purely fictional environment. Sensing devices included interactive devices such as the three-dimensional helmet-mounted display, data gloves, and data clothes worn by the operator, as well as various sensing devices set in the real environment for sensing. The specific activity status of the human body could be obtained through these devices [6]. Menolotto et al. proposed that with the rise of motion capture technology, efficient and fast acquisition of realistic three-dimensional human motion data had become a reality. Motion capture data was successfully used in many fields such as computer animation, video games, and film and television special effects. However, because motion capture was collected based on a specific person and scene, it was inconvenient to reuse the motion data. Therefore, how to analyze, manage, and reuse the existing motion capture data had become a major research focus of current motion capture technology. Reuse methods for motion capture data included motion editing and motion synthesis. Motion editing mainly studied on how to modify a given piece of motion data to make it conform to the new character, new scene, or new constraints set by the user. Motion synthesis took multiple existing three-dimensional human motion data as input, and a new piece of motion data was generated through data processing [7]. Villarreal et al. proposed that with the advent of the era of small ball, the requirements of basketball for athletes' speed, strength, and the outbreak would be further improved. Therefore, it was necessary to seek a scientific and effective training method that was suitable for basketball special sports to adapt to changes in the style of the game. Unilateral training was the most suitable special training method for basketball. On these basis, the integration of compression resistance training could bring about changes to the core strength and lower body strength of athletes that were different from conventional training [8]. Zhao and Liu pointed out that with the rapid development of computer technology, microelectronics technology, simulation system, multimedia sensors, and other technologies and system equipment, VR technology had become an emerging technology that integrates multiple disciplines. Moreover, it was widely used in social development and human life because of its three-dimensional sense, interactivity, immersion, and autonomous sense of substitution. The application of this technology in sports training had effectively improved the efficiency of sports training and strengthened the sports practice ability of athletes. As a common sports event, basketball had attracted much attention from the public for its innovation and optimization of skill teaching and training methods [9]. To sum up, the current VR technology is mature enough to realize many technical problems independently. However, in sports, the application of VR technology is not perfect, especially for the more detailed body motion capture and calculation. Therefore, research is needed to provide technical support for this task to accelerate the application of VR technology in sports and comprehensively promote the development of the sports industry.

The article "Application Effect of Motion Capture Technology in Basketball Resistance Training and Shooting Hit Rate in Immersive Virtual Reality Environment" was published in 2022. Journal: Comput Intell Neurosci.

Based on these, VR technology is first introduced. Then, the motion capture technology is summarized. Finally, the motion capture algorithm is designed and evaluated under basketball resistance training. This work not only provides a technical reference for the improvement of basketball players' shooting percentage but also contributes to the comprehensive development of basketball.

## 2. Research Theories and Methods

### 2.1. Application of VR Technology

VR technology integrates a variety of different types of somatosensory devices to detect and record the real-time behavior of users. It can also analyze the recorded real-time behavior and combine the analysis data with the virtual environment created by the computer. In this way, a virtual environment in which users can interact in real-time in many aspects such as vision, hearing, and touch [10]. Under VR technology, the real environment where the user is located can be any place with little interference. When the user wears the virtual device, all the environment perceived by the user is a virtual effect, which plays an important role in the user's body detection and observation [11].  Figure 1 shows the basic situation of VR technology.

The article "Application Effect of Motion Capture Technology in Basketball Resistance Training and Shooting Hit Rate in Immersive Virtual Reality Environment" was published in 2022. Journal: Comput Intell Neurosci.

From Figure 1, after the user wears the virtual device, the scene presented in front of the user is the scene designed and presented by the computer, and any activities of the user will not produce a scene like the virtual environment in the real environment. The main purpose of VR technology is to simulate and restore the real environment. It virtualizes some things in the real world in the form of symbols to build a virtual world beyond the limitations of the real environment [12]. Humans perceive the environment in the real world through vision, touch, and hearing, and VR technology simulates these perception methods to a great extent. The user's senses can be stimulated through the virtual device, and the user can immerse in the virtual environment and respond to the scene presented in the virtual environment. Also, the user's behavior can be recorded through the device [13]. The virtual devices in the current market mainly simulate the auditory, visual, and tactile senses to construct a virtual world. Meanwhile, the data of the spatial position of the user in the real world is obtained through the positioning device, and the three-dimensional space in the virtual environment is constructed through the computer. The user is integrated into the three-dimensional virtual space through the virtual device. This kind of virtual device greatly improves the user's experience and enables the user to be immersed in it [14]. In addition, the more complex the computer reconstructs the user's location data, the greater the environmental influence the user feels through the virtual device and the better the user's immersion effect. The current VR technology is not mature enough. Because of the influence of factors such as software, hardware, and industry, its application scope is limited. In the future, VR technology will achieve breakthroughs, and it will be applied to face capture, force feedback, character reconstruction, interaction technology, and motion capture [15].

### 2.2. Optimization of Motion Capture Technology

Motion capture technology refers to the technology of acquiring and recording the motion state of the human body. This technology captures and records the motion information data of the human body in space through tracking equipment. It also reconstructs the recorded data on the computer and reproduces the motion state of the human body in the form of the model on the computer [16]. According to the principle of motion capture technology, the technology is divided into mechanical, optical, acoustic, inertial sensor, and electromagnetic.

The article "Application Effect of Motion Capture Technology in Basketball Resistance Training and Shooting Hit Rate in Immersive Virtual Reality Environment" was published in 2022. Journal: Comput Intell Neurosci.

Firstly, the optical motion capture technology relies on the motion trajectory of the optical marker points to capture the motion state of the human body. It pasts the optical marker points on the key parts of the human body and detects the motion track of the optical marker points using multiple cameras. The recorded results are transmitted to the computer. Then, the computer motion trajectories captured by multiple cameras from different angles are calculated. The motion state of the optical representation point is reproduced in the form of a space coordinate point. The calculation process relies on the principle of triangulation to maximize the accuracy of calculation results [17]. There is also an optical capture technology that captures and records body loading in an unmarked form. This method relies on computer vision technology, which captures human motion videos through cameras. The human motion status is analyzed through the AI algorithm combined with computer vision technology. Finally, the calculation result is generated into a depth image to complete the human capture task [18].

Human motion capture technology based on inertial sensors refers to acquiring the motion state of the human body through accelerometers, magnetometers, and gyroscopes. The data of the motion state is obtained by the computer, and the data is constructed into a structure in a three-dimensional space. Finally, the calculated data is mapped to the human skeleton to complete the motion capture technology of the human body [19].

Mechanical motion capture technology refers to the acquisition of the height of the athlete and the data information of various parts of the body and binding sensors of different angles to each joint part of the human body. The data in the sensor is acquired after the human body moves, and the data is recorded. Finally, the body information is combined with the acquired motion data to complete the task of human capture [20].  Figure 2 demonstrates the specific situation of human motion capture technology.

Figure 2 indicates that different human motion capture technologies can complete the task of human motion capture, but different motion capture technologies have different technical means. The advanced VR technology is used to capture the human action state perfectly. The specific operation method is as follows: first, the sensor is installed on the athlete's body. Second, the sensor is linked with the computer. Third, the motion track of the sensor is recorded by the computer, and the recorded result is reproduced by the computer to realize the motion capture of the athlete.

The article "Application Effect of Motion Capture Technology in Basketball Resistance Training and Shooting Hit Rate in Immersive Virtual Reality Environment" was published in 2022. Journal: Comput Intell Neurosci.

### 2.3. Basketball Resistance Training and Shooting Analysis

Resistance training refers to the resistance training of the human body. In the training process, people fight against external forces through their strength to make their body muscles strong and enhance their strength [21]. The most common resistance training exercises include weightlifting and single and parallel bar training. Resistance training is designed to work the muscles of different parts of the athlete. For professional athletes, the purpose of resistance training is to improve the professional motor skills of athletes, such as the agility of football players, the coordination ability of volleyball players, and the balance ability of basketball players [22]. Therefore, when athletes perform resistance training, they can strengthen different parts of the body according to their exercise needs and perform different resistance training based on the muscle structure. More resistance is used for larger muscle groups and less resistance for smaller muscle groups. Athletes can effectively train their bodies while protecting their muscles from injury [23]. Resistance training not only improves athletic performance but also slows down the functional decline, such as muscle aging. Besides, it improves flexibility, balance, and explosiveness and promotes the body's metabolic capacity to achieve the goal of losing weight [24].  Figure 3 reveals the basics of resistance training.

Figure 3 implies that the task of resistance training is to improve athletic ability and provide protection for the health of the human body. The VR technology is used to capture and reproduce the sports state of basketball players to improve their professional athletic ability and shooting percentage. Resistance training is developed for basketball players to improve their professional athletic ability and shooting percentage [25].

## 3. Motion Capture Technology for Basketball Players

Basketball players mainly rely on the movement of arms and legs in the process of exercise. The movement of the human body relies on the connection and cooperation of the bones, tendons, and joints of various parts and completes all the movement processes under the control of the nervous system. Therefore, the key parts of the human body need to be monitored through data to obtain information on human movement [26]. The joint conditions of different parts of the human body under VR technology are shown in Figure 4.

In Figure 4, the numbers represent the different joints of the human body. The joints are located in different parts of the body. There is a connection between these joints, which together contribute to the completion of human movements. In VR technology, the joints of various parts of the human body need to be connected to simulate the motion state of the human body [27]. The main method is to install sensors on the human body and connect the sensors. Human joints are virtually framed on a computer. Then, the motion state of the joints of the human body is captured through the motion trajectory of the sensor. Finally, the actual situation of human movement is evaluated according to the results output by the computer.  Figure 5 displays the specific situation of installing the tracker on the human body.

The article "Application Effect of Motion Capture Technology in Basketball Resistance Training and Shooting Hit Rate in Immersive Virtual Reality Environment" was published in 2022. Journal: Comput Intell Neurosci.

From Figure 5, the data tracked by the tracker can be calculated and analyzed through the human body movement angle to construct the movement process of the human body in the three-dimensional space [28]. The relationship between the human body's torso and the torso-mounted tracker is expressed as follows:

(1) $$\begin{array}{c} q_{b}=q_{a}\times \Delta q_{\text{tab}}. \end{array}$$

In (1), *q*_*b*_ represents the posture of the torso, *q*_*a*_ represents the position state of the tracker, and Δ*q*_*t*_ represents the relative relationship between the tracker and the torso. Δ*q*_*t*_ can be obtained from the predetermined initial states (*q*_*a*0_, *q*_*b*0_) of the torso and tracker according to the following equation:

(2) $$\begin{array}{c} \Delta q_{\text{tab}}=q_{b0}\times {\left(q_{a0}\right)}^{-1}. \end{array}$$

Therefore, the tracking and motion capture of the arms of basketball players can also be calculated in this way.

(3) $$\begin{array}{c} \Delta q_{tes}=q_{e0}\times {\left(q_{s0}\right)}^{-1}. \end{array}$$

In (3), Δ*q*_*tes*_ represents the relative relationship between the arm and its tracker, *q*_*e*0_ represents the initial state of the arm, and *q*_*s*0_ represents the initial state of the tracker. Meanwhile, the state of each part of the torso can be calculated through the following equation:

(4) $$\begin{array}{c} q_{b}=q_{a}\times \Delta q_{tab}=q_{a}\times \left({\left(q_{a0}\right)}^{-1}\times q_{b0}\right). \end{array}$$

Besides, the motion state of the arm can also be calculated in this way.

(5) $$\begin{array}{c} q_{e}=q_{s}\times \Delta q_{tes}=q_{s}\times \left({\left(q_{s0}\right)}^{-1}\times q_{e0}\right). \end{array}$$

The position of the shoulder joint can be expressed as follows:

(6) $$\begin{array}{c} p_{s}=p_{r}\pm T_{R}^{w}\times \frac{1}{2}L_{b}. \end{array}$$

In (6), *p*_*s*_ represents the position state of the shoulder joint, *p*_*r*_ represents the middle part of the thoracic cavity, *L*_*b*_ represents the body width, and *T*_*R*_^*w*^ represents the coordinate system of the thoracic cavity. The position state of the elbow joint is calculated according to the following equation:

(7) $$\begin{array}{c} p_{e}=p_{s}+T_{s}^{w}\times L_{U}. \end{array}$$

In (7), *p*_*e*_ represents the position state of the elbow joint, *T*_*s*_^*w*^ represents the coordinate system of the shoulder joint, and *L*_*U*_ represents the length of the arm. After the state of each joint is vectorized, the vector calculation equation is

(8) $$\begin{array}{c} V_{es}=p_{s}-p_{e},\\ V_{eh}=p_{h}-p_{e}. \end{array}$$

Here, *V*_*es*_ represents the unit vector from the elbow joint to the shoulder joint, *V*_*eh*_ represents the unit vector from the elbow joint to the wrist joint, and *p*_*h*_ represents the position of the wrist joint. Therefore, the angle between two vectors can be calculated by the cosine theorem

(9) $$\begin{array}{c} \alpha_{e}=180^{\circ }-\text{arccos}\left(V_{es},V_{eh}\right). \end{array}$$

In (9), *α*_*e*_ represents the final angle between the human joints. The motion state of the human arm can be captured through the above calculation process. The specific process of motion capture for the human body is revealed in Figure 6.

The article "Application Effect of Motion Capture Technology in Basketball Resistance Training and Shooting Hit Rate in Immersive Virtual Reality Environment" was published in 2022. Journal: Comput Intell Neurosci.

From Figure 6, firstly, the joints of various parts of the human body should be named, and then the tracking equipment needs to be initialized. The initial position of each joint of the human body is located through the wearable device. Finally, a coordinate system is constructed for the joints of the human body, and the movement of the human body reflects the movement process of the body in the coordinate system. Then, the reproduction process of the human motion state in the computer is realized by capturing the data.

## 4. Explanation of Research Data

Basketball players of different heights, genders, and age groups participated in this study, and VR technology was used to capture the process of their shots. Then, the recorded data was analyzed, and the athlete's resistance training process was assessed by shooting tests. The data of the athletes are shown in Table 1.

Table 1 manifests that the athletes studied here are players of a basketball club, with a total of 30 people. Because the best age of current basketball players is between 25- and 32-year-old, this work divides this interval into three subintervals to research athletes of different ages. Athletes of different genders have a large gap in sports status, so athletes are mainly divided according to gender. Moreover, height is one of the important influencing factors of basketball, so it is very important to study the shooting of basketball players according to the height. Basketball players are generally tall, and the height requirements of various basketball leagues are around 200 cm. As a result, athletes are divided according to the general height of basketball players. To sum up, this work performs motion capture on athletes. A 15-day special resistance training is carried out according to their characteristics to evaluate the shooting percentage before and after training.

The article "Application Effect of Motion Capture Technology in Basketball Resistance Training and Shooting Hit Rate in Immersive Virtual Reality Environment" was published in 2022. Journal: Comput Intell Neurosci.

## 5. Basketball Evaluation under Motion Capture

### 5.1. Evaluation of Basic Sports Status of Basketball Projects

In basketball, the physical requirements for players are very high. Athletes need to have agility, stamina, and shooting percentage. These are the basic requirements in basketball, so players need to experience a long period of training such as physical training and shooting training. Resistance training of the body is also crucial for the basketball players.  Figure 7 reveals the basic movement of male and female athletes before training.

From Figure 7, male athletes performed basic training for a maximum of 6 years and a minimum of 2 years before undergoing motion capture and specific resistance training. The largest number of training durations are 4 and 5 years. The longest training period for female athletes is 5 years and the shortest is 2 years. The largest training period is 2 years. Besides, the shooting percentage of male athletes is between 32% and 47%, and that of female athletes is between 28% and 42%.

### 5.2. Evaluation of Motion Capture for Athlete Shots

The most important thing in basketball shooting is the movement of the athlete's arm, and the main role of other body parts is to coordinate and assist the movement of the arm. Therefore, arm movement loading capture and special resistance training for basketball players can improve their shooting percentage. The motion capture results for athletes are shown in Figure 8.

From Figure 8, the shooting action of the basketball player is captured accordingly by capturing the joint motion of the basketball player and calculating the vector position. The results show that the capture method designed here is more perfect for the shooting motion capture of athletes than that of the two-dimensional motion capture technology. It improves the training effect of athletes and helps players to conduct resistance training on themselves, thereby comprehensively promoting their strength.

### 5.3. Evaluation of the Effect of Resistance Training

Resistance training can not only improve the comprehensive physical fitness of professional athletes but also strengthen training to different degrees according to different parts to improve professional athletic ability. The motion capture of VR technology is studied by evaluating the motion state of the basketball players before and after resistance training.  Figure 9 displays the change in shooting percentage of different basketball players before and after resistance training.

The article "Application Effect of Motion Capture Technology in Basketball Resistance Training and Shooting Hit Rate in Immersive Virtual Reality Environment" was published in 2022. Journal: Comput Intell Neurosci.

From Figure 9, the legend in Figure 9(a) represents the age of the athlete, and the legend in Figure 9(c) represents the height of the athlete. Among age-categorized athletes, the most obvious improvement in the shooting percentage across age groups are the athletes aged between 33 and36-year-old, with a maximum shooting percentage improvement of about 14% after resistance training. In the gender categories, female athletes have the highest shooting percentage, while male athletes have the lowest shooting percentage. Finally, in the height categories, athletes with 190–195 cm have the greatest improvement in shooting percentage, which is between 8% and 14%. Athletes with 200–205 cm have the lowest improvement in shooting percentage, generally between 4% and 10%.

## 6. Conclusion

With the development of science and technology, more and more computer technologies have made important contributions to the development of society. As a mainstream project in the current society, promoting its continuous development also plays a vital role in social development. The purpose is to improve the shooting effect of basketball players and facilitate the development of basketball. This work optimizes the resistance training process of basketball players through motion capture technology to improve the shooting rate of basketball players in an immersive VR environment. Firstly, VR technology and motion capture technology are discussed. Then, the basketball resistance training is summarized. Finally, the basketball player's shooting motion state is analyzed based on the motion capture technology, and specific resistance training and shooting percentage assessments are performed through the motion state. Shooting percentage tests are conducted on athletes before motion capture and resistance training, and it is found that athletes' shooting percentages are generally low. The shooting percentage of male athletes is 32%–47%, and that of female athletes is 28%–42%. After motion capture and special resistance training, the shooting state of the athletes is accurately captured. After special resistance training is carried out on the athletes according to the analysis results, it is found that the shooting percentage of the athletes generally increased. The highest shooting percentage increased is about 14%, and the lowest is around 4%. Athletes of different heights have the greatest difference in shooting percentage improvement. Although this work provides a reliable technique for basketball shooting percentage, the training time for athletes is short, and the effect of practical application is not fully demonstrated. Therefore, the research on the practical application effect of this technology will be strengthened in future research.

The article "Application Effect of Motion Capture Technology in Basketball Resistance Training and Shooting Hit Rate in Immersive Virtual Reality Environment" was published in 2022. Journal: Comput Intell Neurosci.

## Figures and Tables

**Figure 1:** Basic situation of VR technology.

**Figure 2:** The specific situation of human motion capture technology.

**Figure 3:** Basic situation of resistance training. (a) Horizontal bar, (b) dumbbell, (c) hula hoop, (d) barbell, (e) jump rope, (f) treadmill, (g) sandbag, (h) balance ball, and (i) sit and push.

**Figure 4:** Joint conditions of different parts of the human body under VR technology.

**Figure 5:** The specific situation of the human body installation tracker.

**Figure 6:** The specific process of motion capture for the human body.

**Figure 7:** Basic sports status of basketball players ((a) the basic training time of the athlete and (b) the shooting percentage of the athlete).

**Figure 8:** The capture results of basketball players by VR technology ((a) is a two-dimensional frame diagram and (b) is the motion capture results of VR technology).

**Figure 9:** Comparison of shooting percentages of basketball players before and after special resistance training ((a) age classification, (b) gender classification, and (c) height classification).

**Table 1:** Data information of athletes.

Classification 1	Classification 2	Number of people	Proportion (%)
Age	25–38	8	26.7
	29–32	10	33.3
	33–36	12	40.0

Gender	Male	15	50.0
	Female	15	50.0

Height (cm)	190–195	6	20.0
	195–200	8	26.7
	200–205	10	33.3
	205–210	6	20.0

## Data Availability

The data used to support the findings of this study are included within the article.
